# Obstacle Capability of an Air-Ground Amphibious Reconnaissance Robot with a Planetary Wheel-Leg Type Structure

**DOI:** 10.1155/2021/7925707

**Published:** 2021-11-18

**Authors:** Enzhong Zhang, Ruiyang Sun, Zaixiang Pang, Shuai Liu

**Affiliations:** School of Mechatronical Engineering, Changchun University of Technology, Changchun, China

## Abstract

According to the requirements of the reconnaissance robot for the ability to adapt to a complex environment and the in-depth study of the obstacle climbing mechanisms, a planetary wheel-leg-combined mechanism capable of adapting to complex terrains is proposed. According to the proposed planetary wheel-leg-combined mechanism, the land part of the air-ground amphibious reconnaissance robot is designed. Considering the obstacle and fast marching performance, four groups of combined wheel-leg mechanisms are adopted in the land bank. Under the action of three kinds of obstacles, the stability and the movement ability of the robot are analyzed by using the static method. The parameter model of the reconnaissance robot is built by a virtual prototype dynamics software MSC.ADMAS. The kinematic characteristic curves of each component and the whole prototype are obtained, which provides a theoretical basis for the design and numerical calculation of the robot structure. Finally, the climbing ability tests of the reconnaissance robot prototype verify the reliability and practicability of the body structure of the reconnaissance robot.

## 1. Introduction

Global economic growth has driven the development and progress of science and technology, and military activities are particularly important. In large- and medium-sized cities that have become targets of various military activities, some cutting-edge technologies are gradually playing an indelible role. Street fighting has become one of the important tasks of the modern army and it is also one of the difficulties of the combat. Reconnaissance is the primary task of urban warfare. Reconnaissance missions are dangerous because urban buildings are dense, tall, and solid; roads are smooth with generally small slopes; a great number of semienclosed structures with less export, and the underground engineering facilities are numerous with complex structures and three-dimensional environments. Thus, unmanned systems have a unique advantage because of its zero casualty, real-time performance, and good concealment [1, 2].

Although unmanned systems have been greatly applied, there are still some drawbacks [3]. For example, the obstacle ability of an army's small ground robot is insufficient and slow, particularly in reconnaissance. The small unmanned aerial vehicle [4, 5] has several problems, such as difficult operation, poor endurance, insufficient ability to monitor the target, and doing continuous reconnaissance. The environment has become a complex battlefield because of the rapid technological development, and existing unmanned systems cannot satisfy the demands. Thus, the development of an air-ground amphibious robot (the robot designed in this paper can move in the air and on the ground but does not involve underwater movement, so its name is an air-ground amphibious robot), which has a certain obstacle climbing capability, is the inevitable development trend in the future. The research on amphibious robots with certain ability of obstacle climbing is more in-depth abroad; the representative one is HyTAQ Robot (hybrid terrestrial and aerial quadrotor, land and air amphibious quadrotor robot), which can move in the air and on the ground. Quadrotor technologies are adopted and the structures are simple. The robot can be operated in ground mode for 27 minutes and move approximately 2400 m. However, the ground movement is inaccurate, which seriously affects its performance [6]. MUWA is a variable pitch quadrotor flying robot for multifield locomotion, that is, standing and rolling at a given tilt angle on the ground like a tire, along with floating and moving on the water surface [7]; the MMALV [8] (morphing micro air-land vehicle) robot is a new type of micro air and land vehicle that can carry out aviation and land movement. It is an integration of power, joint, and leg passive adaptation, which allows it to fly, land, and walk on the ground and over obstacles, etc., so it can be widely applied in different field environments; the “Pegma” deformable land and air amphibious robot [9–11], which can carries a variety of loads, has an endurance of 20 minutes, a maximum travel speed of 4.8 km/h, a maximum flight speed of 84 km/h, and so on. The research on an amphibious robot in land and air that started late in China, especially the amphibious equipment in land and air that can complete vertical takeoff and landing, is few. The ExplorerIII [12], a new amphibious robot developed by the State Key Laboratory, has a total length of 117 cm and a total weight of 6.5 kg, which can complete amphibious movement very well.

The air-ground amphibious robot research started late and has not completed the design of air-ground amphibious VTOL (vertical takeoff and landing) equipment. Therefore, this paper proposes an air-ground amphibious reconnaissance robot with the planetary wheel-leg-type structure. To verify the ground obstacle capability of the robot, a reconnaissance robot obstacle parameter prediction model is constructed based on the ADAMS dynamic simulation software. The centroid displacement, velocity, and relative contact force curve of the robot are simulated with different obstacles, which provide theoretical bases for the design of the mechanism of the reconnaissance robot. The experimental prototypes of the reconnaissance robot have a good obstacle climbing capability, which verify the feasibility and rationality of the structure.

The advantages of this paper can be summarized as follows:

1. The planetary wheel structure is adopted, which allows the designed robot a better ability to overcome obstacles and adapt to the environment and take into account the function of overcoming obstacles and moving fast
2. Static analysis of the obstacle climbing ability under different conditions is carried out to finally determine the obstacle climbing ability, and its reliability is guaranteed
3. The virtual prototype dynamics software MSC.ADAMS is used for analysis to further determine the stability of the prototype

The rest of the paper is summarized as follows. The second part analyzes the mobile mechanism of the robot and further introduces the planetary wheel mechanism on the basis of analyzing the common defects of the mobile mechanism and briefly describes the overall structure and planetary wheel mechanism of the amphibious reconnaissance robot on land and air. In the third part, a suitable motor is chosen according to the size of the actual torque and the detailed parameters of the motor are given. In the fourth part, the stress of the two front wheels and one side wheels is analyzed and the expression form of the vertical obstacle height is finally determined. In the fifth part, the limiting obstacle climbing height of the scout robot is determined by the diagram and the expression is given. In the sixth part, in order to make the scout robot act more smoothly, the obstacle climbing of the scout robot is simulated and analyzed. In the seventh part, a field test is carried out to verify the stability of the robot over obstacles. Finally, the conclusion is given in the eighth part.

## 2. Land Part Structure of the Air-Ground Amphibious Reconnaissance Robot

To adapt to the terrain change in a complex terrain environment, the reconnaissance robot has the more complex structure. Three common structure categories exist: wheeled, crawler type, and leg type [13, 14]. The wheeled mobile robot is fast with flexible control, but the capacity in overcoming obstacles is limited and its adaptability is poor [15, 16]. The crawler-type mobile robot has a good travel mechanism and a large ground contact surface. And, it has a great performance and adaptability to adapt to the terrain change. However, its structure is complex and its volume is large and not flexible enough to turn [17, 18]. The legged mobile robot is highly adaptable, but its control is the most complex [19, 20]. Through the analysis of the motion characteristics of different mobile mechanisms, the motion characteristics of existing robot platforms, and the specific requirements of an air-ground amphibious reconnaissance robot, an amphibious reconnaissance robot planetary wheel–leg-type mobile robot is proposed. It can satisfy multiple requirements in a complex environment, climb over obstacles, and move smoothly in uneven terrains [21]. The robot can change movement patterns according to the terrain by wheel and leg movement combinations, which means using the wheels to achieve high-speed movement and using the legs to improve their ability to adapt to complex terrain environments. Furthermore, it has a compact structure and high efficiency.

Figure 1 is a schematic structure of the air-ground amphibious reconnaissance robot. The land bank is mainly composed of two parts: the main body and four groups of combined wheel-leg mechanisms. The main body has a supporting function, and the main body part is equipped with two brushless motors [22], which drive four groups of combined wheel legs on both sides. Each brushless motor is connected with a synchronous toothed belt wheel and is driven by the meshing of the synchronous toothed belt and the single-side tooth synchronous belt. To reduce the gap in the belt pulley at both ends of the belt and increase the compression of the belt spring, the outside of the belt pulley clamps the pressure synchronous belt in the single tooth to the single tooth synchronous belt tension. When the output shaft of gearbox outputs low speed and high torque, the leg will swing with steering engine to adjust the body height. The structure is shown in Figure 2.

As shown in Figure 1, the wing length of the flying part of the robot is 80 mm and the land part is composed of four planetary wheels. Take a single wheel for analysis, as shown in Figure 2, the diameter of the small wheel is 28 mm, and the vertical distance from the center point of the three small wheels to the ground is 50 mm.

The planetary gear mechanism [23] is mainly composed of the gearbox, gear pawl, main shaft input gear, ratchet, synchronous stepping spur gear, and double-tooth synchronous belt. The power of the planetary wheel is provided by a brushless motor. The robot moves forward with the ordinary wheel when the actuator has a detent movement and synchronous gear output shaft speed and wheel rotation. When the actuator has pawl actuation, the bionic leg function is realized relative to the wheels on the overturned wheel leg side and wheel leg side [24]. The specific structure is shown in Figure 3.

## 3. The Motor Selection

The output torque of the motor is the main factor that determines the ultimate barrier climbing height. When the front wheel of the ground-air amphibious reconnaissance robot is overcoming the obstacle, the overall center of gravity of the robot will move backward and the support force of the ground on the rear wheel will increase with the increase of the elevation angle of the vehicle body. When the front wheel reaches the end of the jump phase, the supporting force is at its maximum and the torque required is also at its maximum.

The mass of the amphibious reconnaissance robot is 4 kg, the dynamic friction coefficient of the wheel is 0.3, the radius of the planetary wheel is 0.014 m, and the obtained required torque after plugging in the actual data is 0.165 N/m. The robot is driven by two motors, so the torque required by each motor is 0.082 N/m. According to the calculated minimum torque [25, 26], the brushless DC motor is selected and the motor parameters are shown in Table 1.

## 4. Two Planetary Wheels Climbing Synchronously

Figure 4 shows a mechanical model of the reconnaissance robot driving when two planetary wheels are climbing synchronously. The following equilibrium equation is obtained by analyzing the robot.

(1) $$\begin{array}{c} N_{1}\sin\alpha +F_{t1}\cos\alpha +\overset{4}{4\sum_{i=2}}N_{i}=G, \end{array}$$

(2) $$\begin{array}{c} N_{1}\cos\alpha -F_{t1}\sin\alpha +\overset{4}{\underset{i=2}{\sum }}F_{fi}-\overset{4}{\underset{i=2}{\sum }}F_{ti}=0, \end{array}$$

(3) $$\begin{array}{c} \frac{D}{2}\overset{4}{\underset{i=2}{\sum }}F_{ti}+G\left(L_{\text{front}}+\frac{b}{2}\right)-N_{2}b-N_{3}L-N_{4}\left(L+b\right)-\frac{D}{2}\overset{4}{\underset{i=2}{\sum }}F_{fi}=0. \end{array}$$

The reaction force on front planetary wheel 1 is *N*_1_ in the formula; *N*_2_, *N*_3_, and *N*_4_ are the ground reaction forces of wheels 2, 3, and 4, respectively; *G* is the weight of the air-ground amphibious reconnaissance robot; *D* is the diameter of the wheel on the planet; *b* is the distance between the centers of two wheels that land simultaneously in the planetary gears; *L*_front_ is the air-ground amphibious reconnaissance robot centroid before the planetary wheel center distance; *F*_*t*1_ is the driving force of round 1 of negotiation; *F*_*t*2_, *F*_*t*3_, and *F*_t4_ are the horizontal driving forces of wheels 2, 3, and 4, respectively; *F*_*f*2_, *F*_*f*3_, and *F*_*f*4_ are the rolling resistances of wheels 2, 3, and 4, respectively. Meanwhile,

(4) $$\begin{array}{c} F_{fi}=f\cdot N_{i},\;\left(i=2,3,4\right), \end{array}$$

where *f* is the rolling resistance coefficient.

In the process of planetary wheel over the obstacle, wheel 1, wheel 2, wheel 3, and wheel 4 are driven by the same brushless motor, so the torque is evenly distributed and the adhesion coefficient *φ* of wheels 1 and 2 are the same, which is

(5) $$\begin{array}{c} F_{t1}=F_{t2}=\min\left(N_{1},N_{2}\right)\cdot \varphi , \end{array}$$

In order to obtain the vertical height (*h*_*s*_)_1_ that the two front wheels can climb over when they cross the obstacle at the same time, assuming that the vertical force acting on wheel 1 and wheel 2 and the horizontal driving force acting on the front and rear axles are equal, then, in general road conditions,

(6) $$\begin{array}{c} f=0, \end{array}$$

(7) $$\begin{array}{c} N_{1}\sin\alpha +F_{t1}\cos\alpha =N_{2}, \end{array}$$

(8) $$\begin{array}{c} F_{t3}+F_{t4}=F_{t2}+F_{t1}\sin\alpha -N_{1}\cos\alpha . \end{array}$$

According to the actual situation, the force can be divided into two situations:

1. When *N*_1_ < *N*_2_,

(9) $$\begin{array}{c} N_{2}=N_{1}\sin\alpha +N_{1}\cdot \varphi \cos\alpha . \end{array}$$

Substituting equations (6) and (9) into the second equation in equation (1) and taking into account *F*_*t*1_ = *F*_*t*2_ = *N*_1_ · *φ*, the solution is:

(10) $$\begin{array}{c} \cos\alpha =\varphi +\varphi \sin\alpha \end{array}$$

(2) When *N*_1_ > *N*_2_,

(11) $$\begin{array}{c} N_{2}=N_{1}\sin\alpha +N_{2}\cdot \varphi \cos\alpha \end{array}$$

Therefore, the following equation can be obtained:

(12) $$\begin{array}{c} \frac{N_{2}}{N_{1}}=\frac{\sin\alpha }{1-\varphi \cos\alpha }. \end{array}$$

Substituting equations (6) and (11) into the second equation in equation (1) and taking into account *F*_*t*1_ = *F*_*t*2_ = *N*_2_ · *φ*, the solution is

(13) $$\begin{array}{c} \frac{N_{2}}{N_{1}}=\frac{\cos\alpha }{\varphi +\varphi \sin\alpha }. \end{array}$$

Simultaneously, equation (14) can be obtained combining equations (12) and (13):

(14) $$\begin{array}{c} \cos\alpha =\varphi +\varphi \sin\alpha . \end{array}$$

Therefore, the obstacle climbing ability of the reconnaissance robot can be expressed regardless of the situation. Finally, from the mechanics relation in Figure 4, the following solution is obtained:

(15) $$\begin{array}{c} \sin\alpha =1-2\frac{h}{D}. \end{array}$$

Equation (15) is substituted into equation (14) and results in the following solution:

(16) $$\begin{array}{c} {\left(h_{s}\right)}_{1}=\frac{\varphi^{2}}{\varphi^{2}+1}\cdot D. \end{array}$$

Therefore, if the vertical obstacle of the two front wheels and the obstacle height are less than (*h*_*s*_)_1_, the planetary wheel does not need to be flipped. If the vertical barrier height is more than (*h*_*s*_)_1_, the planetary wheel needs to be turned over to get over the vertical obstacle.

## 5. Single-Planetary Wheel Obstacle

The road condition is changeable in the process of reconnaissance. The single-planetary wheel case cannot be avoided. Thus, establishing the mechanical model of a single planetary wheel is necessary. The stress analysis is shown in Figures 5 and 6. The following equations are obtained through the robot balance analysis.

(17) $$\begin{array}{c} N_{1}\sin\alpha +F_{t1}\cos\alpha +\overset{5}{\underset{i=2}{\sum }}N_{i}=G, \end{array}$$

(18) $$\begin{array}{c} N_{1}\cos\alpha -F_{t1}\sin\alpha +\overset{5}{\underset{i=2}{\sum }}F_{fi}-\overset{5}{\underset{i=2}{\sum }}F_{ti}=0, \end{array}$$

(19) $$\begin{array}{c} \frac{D}{2}\overset{5}{\underset{i=1}{\sum }}F_{ti}+G\left(L_{\text{front}}+\frac{b}{2}\right)-N_{2}b-N_{4}b-N_{5}\left(L+b\right)-\frac{D}{2}\overset{5}{\underset{i=2}{\sum }}F_{fi}=0. \end{array}$$

The reverse acting force on right planetary wheel 1 is *N*_1_ in the formula; *N*_2_, *N*_3_, and *N*_4_ are the ground reaction force of wheels 2, 3, and 4, respectively; *N*_5_ is the rear axle load.

When the obstacle is in front of the planetary gear, wheels 1 and 2 are driven by the same brushless motor and *φ* is the same, thus obtaining

(20) $$\begin{array}{c} F_{ti}=F_{t2}=\min\left(N_{1},N_{2}\right)\cdot \varphi . \end{array}$$

Similarly, assuming that the road conditions are generally good,

(21) $$\begin{array}{c} f=0, \end{array}$$

(22) $$\begin{array}{c} N_{1}\sin\alpha +F_{t1}\cos\alpha =N_{2}, \end{array}$$

(23) $$\begin{array}{c} F_{t2}+F_{t1}\sin\alpha -N_{1}\cos\alpha =F_{t3}+F_{t4}, \end{array}$$

(24) $$\begin{array}{c} F_{t1}\sin\alpha -N_{1}\cos\alpha +F_{t2}+F_{t3}+F_{t4}=F_{t5}. \end{array}$$

1. When *N*_1_ < *N*_2_,

(25) $$\begin{array}{c} N_{2}=N_{1}\sin\alpha +N_{1}\cdot \varphi \cos\alpha . \end{array}$$

Substituting equations (21) and (25) into the second equation in equation (17) and taking into account *F*_*t*1_ = *F*_*t*2_ = *N*_1_ · *φ*, the solution is

(26) $$\begin{array}{c} \cos\alpha =\varphi +\varphi \sin\alpha \end{array}$$

(2) When *N*_1_ > *N*_2_,

(27) $$\begin{array}{c} N_{2}=N_{1}\sin\alpha +N_{2}\cdot \varphi \cos\alpha . \end{array}$$

Therefore, the following equation can be obtained:

(28) $$\begin{array}{c} \frac{N_{2}}{N_{1}}=\frac{\sin\alpha }{1-\varphi \cos\alpha }. \end{array}$$

Substitute equations (21) and (27) into the second equation in equation (17) and taking into account *F*_*t*1_ = *F*_*t*2_ = *N*_2_ · *φ*, the solution is

(29) $$\begin{array}{c} \frac{N_{2}}{N_{1}}=\frac{\cos\alpha }{\varphi +\varphi \sin\alpha }. \end{array}$$

Simultaneously, equation (30) can be obtained combining equations (28) and (29):

(30) $$\begin{array}{c} \cos\alpha =\varphi +\varphi \sin\alpha . \end{array}$$

Thus, it can be known that the height of vertical obstacle overcame by a single planetary wheel (*h*_*s*_)_2_ can be expressed by equation (30) in any case. Substituting equation (15) into (30) obtains the solution

(31) $$\begin{array}{c} {\left(h_{s}\right)}_{2}=\frac{\varphi^{2}}{\varphi^{2}+1}\cdot D. \end{array}$$

From the above theoretical results, the reconnaissance robot has the ability to overcome the vertical barrier consistently regardless of the situation.

## 6. Limiting the Vertical Obstacle Height of the Reconnaissance Robot

When the planetary wheel encounters a vertical obstacle height more than (*h*_*s*_)_*i*_, it will need to turn over the planetary wheel to overcome the obstacle. The limiting value of the vertical barrier *H*_max_ can be expressed in the following formula:

(32) $$\begin{array}{c} H_{\max}<=\frac{D}{2+\left(2R\sin60^{{}^{\circ}}\right)}, \end{array}$$

where *R* represents the torque of the planetary wheel.

## 7. ADAMS-Simulated Analysis

### 7.1. Planetary Wheel Encounters Vertical Obstacle

For robot development, there are corresponding tests in every stage from concept to requirement and from design to implementation and virtual tests realized by simulation modeling can optimally adjust parameters. In this paper, when the obstacles are 8 mm and 80 mm, the obstacle crossing test can reduce the number of prototype tests and know the obstacle crossing limits in both cases, thus creating a prerequisite for the smooth operation of the robot.

Figure 7 shows the simulation model of the two planetary wheels climbing the vertical obstacle simultaneously. *φ* is assumed to be 0.6 between the wheel and the ground. By continuously changing the height of the parameterized obstacle model, the analysis and simulation results are listed as follows:

1. When the height of a vertical obstacle (*h*_*s*_)_*i*_ ≤ 8mm, the planetary wheel can move pass the obstacles
2. When the height of a vertical obstacle (*h*_*s*_)_*i*_ > 8mm, the planetary wheel cannot move pass the obstacles

Meanwhile, *φ* = 0.6 is substituted in the theoretical formulas to obtain the maximum obstacle climbing height of 7.41 mm. Compared with the simulation result, the relative error is 7.96%. Many assumptions about the *φ* are made, and the simulation results are compared with the theoretical ones. The errors are all below 10%. The results show that the above theoretical inference process is reliable and the model is feasible.

### 7.2. Limiting Height of Vertical Obstacle Climbing

Figure 8 shows the simulation model of the limiting vertical overcoming of the reconnaissance robot, by continuously changing the height of the parametric obstacle model, the following simulation results are obtained:

1. When the height of the vertical obstacle *h* ≤ 80mm, the reconnaissance robot can move pass the obstacles
2. When the height of the vertical obstacle *h* > 80mm, the reconnaissance robot cannot move pass the obstacles

Meanwhile, each known values are substituted in the theoretical formulas to calculate the maximum obstacle climbing height of 83.28 mm. Compared with the simulation result, the relative error is 3.94%. So, the derivation process is rigorous, the theory and the practice are reliable, and the model is feasible.

### 7.3. Stability Analysis of the Reconnaissance Robot Getting over the Obstacles

When the reconnaissance robot successfully overcomes vertical obstacles at different heights and in different conditions, the kinematics curves of the main vehicle body is shown in Figure 9. They represent the position and pose changes of the main vehicle body when the reconnaissance robot is getting over the obstacle without any control under the external load. The change of position coordinates of the mass center decreases with the increase of time. The contact force between the planetary wheel and the ground is stable with the increase of time. The mass acceleration fluctuates wildly within a certain interval and reaches a plateau. Thus, the stability of the reconnaissance robot is verified during obstacle climbing.

For a rigid body, if the mass of each component and the position of the centroid point in a unified coordinate system can be known, the total position of the centroid point of the rigid body in the coordinate system can be calculated by the following formula:

(33) $$\begin{array}{c} x=\frac{\sum_{i=1}^{k}m_{i}x_{i}}{\sum_{i=1}^{k}m_{i}},\\ y=\frac{\sum_{i=1}^{k}m_{i}y_{i}}{\sum_{i=1}^{k}m_{i}},\\ z=\frac{\sum_{i=1}^{k}m_{i}z_{i}}{\sum_{i=1}^{k}m_{i}}. \end{array}$$

Through the calculation of the program, when the active driving angle of the robot changes once during obstacle crossing, the posture, center point position, and total centroid position of the robot will be recorded and the total centroid position will be drawn into an image for direct output, as shown in Figure 9(a).

In the process of obstacle surmounting, the position of the center of mass of the robot changes due to terrain factors. The centroid determines the performance of obstacle crossing, and the motion attitude affects the position of the centroid. The change of the position of the centroid changes some values, which leads to the fluctuation of the centroid acceleration in a certain range.

The obstacle crossing height simulated in this test is 80 mm.

## 8. Test of the Sample Equipment

The overstepping ability of the air-ground amphibious reconnaissance robot, the fast movement on irregular terrain, the overstepping of the two planetary wheels simultaneously, and the overcoming of an obstacle by a single planetary wheel are shown in Figure 10. The speed of the fast movement on an irregular terrain, cement pavement, and cotta road with 80 mm/s is chosen. The result of the experiment validates that the robot can move smoothly and meet the requirements of smooth obstacle climbing. The two planetary wheels can overcome the vertical obstacle with a height of 20 mm simultaneously. They smoothly overcome the steps. The single planetary wheel can overcome the vertical obstacle of cotta with a height of 54 mm. It smoothly overcomes the obstacle. The experiment shows that reconnaissance robot is suited for various types of the environment and possesses flexible motion behaviors, excellent kinetic characters, and off-road abilities.

## 9. Conclusion

This paper presents a planetary wheel-legged air-ground amphibious reconnaissance robot. To verify the terrain adaptability and obstacle climbing capability of the robot, the parameters of the obstacle prediction model of the reconnaissance robot are obtained based on the dynamic simulating software MSC.ADAMS. Simulation research is performed under various obstacle conditions, and the starting curves of the displacement of the mass center, velocity, and contact pressure are plotted online. The results provide the theoretical bases for the design of the mechanical system of the reconnaissance robot.

The planetary wheel legged reconnaissance robot designed in this paper can climb only the same vertical height as when the wheels encounter obstacles *φ* and *D*, independent of other parameters of the reconnaissance robot. In addition, from the theoretical derivation results, whether two front wheels cross the obstacle at the same time or a single wheel, the ability to climb the vertical obstacle is the same in these two cases. The simulation analysis of software MSC.ADAMS shows that the theoretical derivation is reliable.

When the height of the vertical obstacle is greater than the height of the vertical obstacle that can be climbed, the wheels need to turn over to cross the vertical obstacle and the limit height of the vertical obstacle that can be crossed is given through theoretical calculation, which makes the article more convincing. Finally, the structure is rational and feasible based on the prototype fabrication and good obstacle performance of the reconnaissance robot.

In future work, the structure optimization will be conducted to make the robot more compact. By optimizing the structure of the reconnaissance robot, it can better carry out the reconnaissance operation and adapt to a variety of road conditions and environments. In addition, using more accurate control algorithm can better improve the control accuracy and interaction ability of the robot and improve its operation ability in different environments. The disadvantage is that it takes a lot of time and high cost to adopt the more accurate control algorithm and compact fuselage structure, which is undoubtedly very extravagant when there are no important tasks.

In addition, the control algorithm of the robot will be extensively investigated to enhance the control precision and interaction ability of the robot system. In the process of solving the above shortcomings, a better control system can be designed. In the newly designed control system, infrared and other better sensors (ultrasonic, CCD, etc.) are used to obtain the main data. The virtual prototype model established by a computer for simulation can optimize the obstacle crossing performance or get a structural scheme with better comprehensive performance. The relationship between the tire and the ground is introduced to make the simulation closer to the real situation, and then, the structural dimensions with excellent performance are designed.

## Figures and Tables

**Figure 1:** Schematic structure of air-ground amphibious reconnaissance robot.

**Figure 2:** Main body of the specific structure.

**Figure 3:** Specific structure of the planetary wheel.

**Figure 4:** Mechanical model of the two front planetary wheels at the same time in the case of vertical obstacle balance.

**Figure 5:** Mechanical analysis of planetary gears without obstacles.

**Figure 6:** Mechanical analysis of a single planetary wheel in the case of vertical obstacles.

**Figure 7:** Simulation model of two planetary wheels over the steps at the same time.

**Figure 8:** Limiting vertical obstacle model.

**Figure 9:** Kinematics curves of the main vehicle body.

**Figure 10:** Experiment verifying the robot's overstepping ability.

**Table 1:** Brushless DC motor parameters.

Model	Rated power	Nominal torque	Rate speed	Nominal voltage	Rated current	Short-time overload multiple	Weight	Boundary dimension
Unit	W	N·m	r/min	V	A		kg	mm
45ZW05	14	0.09	1500	12	2	2	0.52	45 × 84

## Data Availability

The data is available by the corresponding email or the correspondence author email.
